# An Improved YOLOX Algorithm for Forest Insect Pest Detection

**DOI:** 10.1155/2022/5787554

**Published:** 2022-08-23

**Authors:** Jiyu Huang, Yong Huang, Hongliang Huang, Weirong Zhu, Jun Zhang, Xiaolong Zhou

**Affiliations:** ^1^Anji County Forestry Bureau, Anji 313300, China; ^2^Zhejiang Forestry Technology Promotion Station, Hangzhou 310020, China; ^3^College of Electrical and Information Engineering, Quzhou University, Quzhou 324000, China

## Abstract

A large number of insect pests in the forest will seriously affect the construction of forest resources and agriculture in China. In this regard, in order to deeply understand and analyze the existing forest pest detection technology, it is found that it cannot meet practical needs. In order to prevent the harm caused by forest pests, it is necessary to correctly identify the types of pests and take targeted control measures. Therefore, this paper proposes a forest pest detection algorithm based on improved YOLOX. Firstly, aiming at the problem that there are few image data of real deep forest pests in the wild, we use Mosaic, Mixup, and random erasure data enhancement to preprocess the images. Secondly, in order to extract fine-grained features, shallow information is introduced into the existing network architecture, and a two-way cross-scale feature fusion mechanism is adopted. Finally, the improved YOLOX algorithm proposed in this paper has achieved the best results on the public forest pest dataset IP102.

## 1. Introduction

Forest resources in many parts of China are being attacked by diseases and insect pests. According to official statistics, there are more than 8000 kinds of forest diseases and insect pests in China. Not only is the coverage area of forest diseases and insect pests broad, but also its growth rate is accelerating in the form of acceleration. It has been difficult to limit forest diseases and insect pests with general pesticides. Coupled with the super reproductive ability of insects and the impact of a large number of human production activities, forest diseases and insect pests have become a major challenge to China's forest resources.

A large number of diseases and pests in forests will seriously affect the construction of forest resources and forest agriculture in China. If diseases and pests are not controlled, the normal growth of forest vegetation will be seriously affected, further causing soil erosion and affecting air quality. The villagers who live in forest agriculture will also suffer huge economic losses. Therefore, it is of great significance to construct forest resources and monitor forest pests and diseases to realize the sustainable development of China's ecological environment.

Compared with traditional monitoring methods, the use of UAVs for forest pest control has the following advantages. First of all, traditional monitoring methods usually invest a lot of human and material resources to go deep into the forest to obtain entity data for analysis but often cannot fully reflect the actual situation of a forest. The experimental object has great particularity, and the UAV can use many technologies in the survey and detection of forest diseases and pests, such as remote sensing and visible light scanning, to clearly grasp the forest health status in the regional area. The real situation of the forest can be accurately located and reflected with less manpower and material resources so that pest control can be carried out accurately. Secondly, the traditional monitoring methods are limited by traffic conditions and are difficult to go deep into remote or harsh areas such as mountains, dense forests, and steep mountains. They are often disturbed by external factors. The application of UAV monitoring can reduce manual operation. These outdoor working environments are difficult and dangerous, and the use of UAV monitoring can go deep into these places and improve the utilization efficiency of human resources. Finally, the timeliness of traditional monitoring methods is not high, and they cannot reflect the situation of the monitored area in real time. Traditional monitoring methods are difficult to ensure the timeliness of data. It takes a lot of time to analyze the data and explore the surrounding terrain, and the real-time situation of the damaged wood cannot be continuously updated. However, the use of UAV technology can better grasp the changes of pests, synchronize the data with the corresponding departments, help people grasp the real situation of diseases and pests timely and accurately, and improve the timeliness of the data.

Traditional pest detection and identification work first rely on hand-made features, including SIFT [1], LBP [2], ORB [3], Color [4], and SURF [5] operators to represent targets. Then, machine learning is used for target recognition, such as support vector machine (SVM) [6], nearest neighbor -K(KNN) [7], random forest [8], and so on. These feature-based methods rely too much on the characterization of feature operators. It lacks robustness to illumination, occlusion, complex environment, and interference of similar targets.

Therefore, the overall classification accuracy is poor. With the excellent performance of deep learning in various fields, it has also attracted the attention of forest pest researchers and introduced it into the detection and identification of pests. Wang et al. [9] proposed a convolution neural network based on the inception module and extended convolution for plant pest identification. Cheng et al. [10] designed a pest identification method using deep residual learning. Compared with the support vector machine and traditional BP neural network, the accuracy of pest image recognition under complex farmland backgrounds is significantly improved. Huang et al. [11] proposed to classify eight categories of tomato pests based on the Convolutional Neural Network (CNN) model and used transfer learning to reduce training time. Liu et al. [12] constructed two migration strategies for pest identification in the Convolutional Neural Network (CNN) through a graph-based visual significance enhancement dataset, combined with migration learning and fine-tuning. However, the above methods are limited by the small dataset, which is easy to lead to the knowledge limitation and overfitting of model learning. In addition, the extracted features are too simple and not robust, and the generalization ability in the actual scene is insufficient.

With the advancement of deep learning technology, many detectors based on convolutional neural networks are now playing a good detection effect. With the advancement of deep learning technology, many detectors based on convolutional neural networks are now playing a good detection effect. The one-stage detectors [12‐15] predict the class and location of the object directly by convolutional neural networks, while faster R-CNN [16] and spare R-CNN [17] are used to generate region proposal by region proposal networks and then perform classification and regression tasks, which is more accurate. The transformer-based detectors [18‐20] have no anchor constraints and no nonextreme value suppression postprocessing step. The end-to-end implementation greatly simplifies the object detection pipeline.

Aiming at the above two problems, this paper proposes a forest pest detection algorithm based on improved YOLOX. For this paper, the main contributions are as follows:

1. Aiming at the problem that there are few image data of real deep forest pests in the wild, after Mosaic and MixUp, random erasing data enhancement is applied to the training data.
2. In order to extract fine-grained features, shallow information is introduced into the existing network architecture, and a two-way cross-scale feature fusion mechanism is adopted.
3. The improved YOLOX algorithm proposed in this paper has achieved the best results on the public forest pest dataset IP102.

## 2. Related Work

### 2.1. Pest Identification Based on Machine Learning

As mentioned above, pest recognition based on the traditional learning method includes two steps: feature extraction and model training. Feature extraction is to extract important related features such as texture, color, and shape of an insect image for target representation. Hassan et al. [12] designed an intelligent insect classification system based on shape and color features to identify grasshoppers and butterflies. The HOG feature was first used in pedestrian detection [21] and gained attention due to its good performance, which was subsequently applied to insect detection by Shen [22] et al. At the same time, Liu et al. [23] also used HOG's maximum stable extreme region (MSER) algorithm for reference to detect aphids with different colors and densities in wheat fields. By extracting HOG features from positive and negative training samples of aphids, the accuracy of aphid detection is improved. Huang et al. [24] used KNN to identify insects. Rani et al. [25] applied an SVM classifier to identify whiteflies, aphids, and thrips in leaf images. Although traditional machine learning can make some achievements in the specific scene, it relies too much on manual feature extraction, is not robust enough, and lacks generalization ability. So, it cannot adapt to scene migration.

### 2.2. Pest Identification Based on Deep Learning

Traditional machine learning relies too much on manual skills in feature extraction and lacks the good fitting ability to data. Compared with machine learning, in recent years, deep learning has become more and more popular. It extracts data features through a Convolutional Neural Network (CNN) for end-to-end training. Its lightweight model and powerful generalization ability have a good performance in subordinate tasks such as target tracking and image recognition. Therefore, the application of deep learning to pest identification has gradually become the current mainstream research hotspot. For example, on the basis of traditional CNN, Chen et al. [10] established a new CNN model for pest identification and tested 550 pictures of 10 categories under natural background, with an accuracy of about 99.67%. Alves et al. [26] designed a new deep residual learning model, which added a seven-layer network and achieved 98% classification accuracy on 1600 common cotton pest datasets. Sun et al. [27] used the JFT-300M dataset and found that there was a logarithmic relationship between the performance of visual tasks and the amount of training data. In China, in order to solve the problem that deep learning is difficult to migrate to agricultural scenes, Kong et al. [28] put forward a multi-stream Gaussian probability fusion network (MPFN), which trained 122,000 images of 181 kinds of pests and diseases and achieved an average recognition accuracy of 93.18%. Yang et al. [29] further optimized the neural network and combined it with the GrabCut algorithm to realize the accurate identification and location of tea garden pests. Although the current pest identification methods based on deep learning have made some achievements, the extracted features are not robust enough because of the single network structure.

## 3. The Proposed Method

The current pest identification methods are limited by the small dataset, which easily leads to the knowledge limitation and overfitting of model learning. In addition, the extracted features are too simple and not robust enough. The generalization ability of actual scenes is insufficient. In view of the above two problems, this paper takes YOLOX [14] as the framework and improves it to deal with the task of forest pest detection.

YOLOX, one of the most accurate detectors available, uses a more efficient data enhancement approach to preprocess the data. It is also an anchor-free frame-based detector, avoiding the problem of unbalanced positive and negative samples with the anchor frame approach. The simultaneous use of decoupled heads for classification and regression tasks is significantly better than other detectors in terms of accuracy and speed. So, we used YOLOX as our baseline and made some improvements.

Firstly, aiming at the problem that there are few pictures of real deep forest pests in the field, after Mosaic and Mixup, random erasing data enhancement is carried out on the training data to prevent overfitting in the process of model training. Secondly, in order to extract fine-grained features, shallow information is introduced into the existing network architecture, and a two-way cross-scale feature fusion mechanism is adopted.  Figure 1 shows the overall framework of the algorithm in this paper.

### 3.1. Data Enhancement

This paper uses Mosaic and Mixup as basic data enhancement. Mosaic data enhancement: four images are spliced by random scaling, random clipping, and random arrangement, which enriches the background and small targets of the detected objects. Mixup data enhancement: overlapping two pictures together can reduce the memory of wrong labels and enhance robustness. The random erased images can improve the robustness against image noise, e.g., partial occlusions and imperfect detections. The effect of the data enhancement is shown in Figure 2.

### 3.2. Backbone

CSPDarknet-53 is used as the backbone network for feature extraction, which consists of five parts: stem, dark2, dark3, dark4, and dark5. Compared with the traditional ResNet-50 network, this backbone not only ensures accuracy but also keeps the system lightweight, and its structure is shown in Figure 3. Each module is described as follows:

1. **Focus module:** Slice an image by taking a value for each pixel at an interval (similar to adjacent down sampling). As a result, the information from W and H is integrated into the channel space. The output channel is expanded by four times. Compared with the original RGB three-channel mode, the spliced image becomes 12 channels. Increasing the number of channels is beneficial to the later calculation, as shown in Figure 4.
2. **CBL module:** It mainly includes three operations: convolution, normalization, and activation function. The specific structure is shown in Figure 5.
3. **SPP module:** Referring to the idea of spatial pyramid pooling, the pooling layer composed of three convolution kernels (5 × 5, 9 × 9, 13 × 13) with different sizes realizes the fusion of local features and global features and enriches the expression ability of the final feature map, as shown in Figure 6.

### 3.3. Improved Neck

Inspired by BIFPN [30], this paper proposes an algorithm for the multiscale fusion of outputs of backbone networks dark2, dark3, dark4, and dark5. In order to extract more robust fine-grained features, this paper proposes an algorithm that considers shallow information in the original framework and further introduces dark2, which is beneficial to small target detection. The BIAFPN structure is a top-down fusion, transferring deep semantic information back to the shallow layer, and then a bottom-up fusion to enhance location information. On this basis, cross-scale fusion is added to the algorithm in this paper (as shown in Figure 7). For each fusion, adaptive weight SUM is added, and the adaptive adding formula is as follows:

(1) $$\begin{array}{c} P_{i+2}^{td}=\text{Conv}\left(\frac{w_{1}\cdot P_{i+2}^{in}+w_{2}\cdot \text{Resize}\left(P_{i+3}^{in}\right)}{w_{1}+w_{2}+\epsilon }\right). \end{array}$$

Here, *i* = {1, 2}; *w*_1_ and *w*_2_ are initialized to 1, *P*_*i*_^*in*^ and *P*_*i*+1_^*in*^ are outputs of corresponding layers of the main network; Conv (.) is usually a convolutional op for feature processing. Resize (.) is the sampling operation to keep the size of the feature map consistent; *ϵ*=0.0001 is a hyperparameter to prevent the divisor from being 0.

(2) $$\begin{array}{c} P_{2}^{\text{out}}=\text{Conv}\left(\frac{w_{1}\cdot P_{2}^{\text{in}}+w_{2}\cdot \text{Resize}\left(P_{3}^{td}\right)}{w_{1}+w_{2}+\epsilon }\right),\\ P_{5}^{\text{out}}=\text{Conv}\left(\frac{w\cdot P_{5}^{\text{in}}+w_{2}\cdot \text{Resize}\left(P_{4}^{\text{out}}\right)}{w_{1}+w_{2}+\epsilon }\right), \end{array}$$

where *w*_1_ and *w*_2_ are initialized to 1 and are normalized to be a probability with a value ranging from 0 to 1, representing the importance of each input.

(3) $$\begin{array}{c} P_{j}^{\text{out}}=\text{Conv}\left(\frac{\mu_{1}\cdot P_{j}^{\text{in}}+\mu_{2}\cdot P_{j}^{td}+\mu_{3}\cdot \text{Resize}\left(P_{j-1}^{\text{out}}\right)}{\mu_{1}+\mu_{2}+\mu_{3}+\epsilon }\right), \end{array}$$

where *j* = {3, 4}; *μ*_1_, *μ*_2_, and *μ*_3_ are initialized to 1 and are normalized to be a probability with a value ranging from 0 to 1, representing the importance of each input. After each fusion, the spatial information and channel information are enhanced by CBAM [31], and finally, the output is obtained. This fusion module can be repeated *n* times. The model diagram of the neck is shown in the middle of the neck module in Figure 7. The calculation of fusion is summarized in Algorithm 1.

### 3.4. Head

As shown in Figure 8, the head section consists of four prediction heads, each with separate classification and regression branches, spliced along the channel, and a reshape operation to multiply W and H. The last 4 prediction heads are spliced along W*∗*H, then each part of the loss is calculated, and the following is the structure diagram of our head part of the model Figure 9.

(1) Decoupled head. It is a well-known problem that classification tasks and regression tasks will conflict, so we put forward the idea of calculating classification tasks and regression tasks separately. The specific structure as shown in the experiment proves that it can improve the accuracy. We understand that the classification task is different from the regression task in terms of focus and interest. The classification task pays more attention to which of the extracted features is closest to the existing categories, while the regression task pays more attention to the position coordinates of the real box so as to correct the boundary box parameters. If a feature map is classified and regressed, the effect will be bad.
(2) Anchor free. At present, most detection algorithms are under an anchor-based architecture, which has the following disadvantages: unbalanced positive and negative samples and more superparameters (anchor number, size, aspect ratio). The model adopts an anchor-free strategy. Each grid only produces one prediction box, and its performance is comparable to that of an anchor-based strategy.
(3) SiamOTA. For the label allocation strategy, we first calculate the cost of the matching degree according to the formula:
  (4) $$\begin{array}{c} c_{ij}=L_{ij}^{cls}+\lambda L_{ij}^{reg}, \end{array}$$
where *L*_*ij*_^*cls*^ and *L*_*ij*_^*reg*^ represent the classification loss and regression loss between the true value and the predicted value, and *λ* is the matching coefficient. We then choose the first *k* minimum cost as a positive sample, and the rest of the predictions are negative samples. *Siam*OTA not only reduces the training time but also avoids additional superparameters.

### 3.5. Loss Function

We calculate classification loss and target score loss by using the binary cross-entropy loss function:

(5) $$\begin{array}{c} \text{BCELoss}=-\left(y\;\log\left(p\left(x\right)\right)+\left(1-y\right)\log\left(1-p\left(x\right)\right)\right), \end{array}$$

where *y* indicates whether it is category information or target, and the value is 1 or 0; *p*(*x*) is the score of each category and the predicted score.

We then calculate the frame loss, predict the frame information, and calculate the IOU(IntersectionofUnion) based on the real frame information calculated by the label. IOU is the intersection ratio between the prediction frame and the real frame, and the prediction frame with a high IOU value can be obtained through NMS postprocessing.

(6) $$\begin{array}{c} \text{IOULoss}=1-\frac{I\left(\tilde{B},B\right)}{U\left(\tilde{B},B\right)}, \end{array}$$

where $\tilde{B}$ is the ground truth, *B* is the prediction box, $I\left(\tilde{B},B\right)$ is the area where the real box and the prediction box intersect, and $U\left(\tilde{B},B\right)$ is the area where the real box and the prediction box merge. The lower the IOULoss value is, the more accurate the prediction is.

## 4. Experimental Results and Analysis

### 4.1. Dataset

The dataset selected for this experiment is IP102 (a large benchmark dataset for pest identification) [32], which has 102 categories and contains 18,981 pictures. The training data and testing data of this experiment are divided into datasets according to 7 : 3. The data display is shown in Figure 10.

### 4.2. Experimental Environment

Python3.7 and Pytorch1.9.1 are used in the experiment, and the model of the graphics card is 2*∗*3090Ti, which is matched with CUDA11.4.

### 4.3. Network Parameter

In order to be transplanted to handheld devices in the later stage, this experiment adopts the YOLOX_S version of the model (the minimum number of parameters). The weights are added, which have been trained on the COCO dataset as pretraining weights. A total of 250 training sessions have been conducted. The first five training sessions are warmed up using the random gradient descent (SGD) algorithm. The learning rate is set as lr = lr_0_ × BatchSize/64, where lr_0_ = 0.01 denotes the initial learning rate, BatchSize = 16 represents that we use this BatchSize during the training, and the learning rate adjustment strategy is cosine annealing.

### 4.4. Contrast Result

In order to verify the effectiveness of the improved YOLOX algorithm proposed in this paper in the task of forest pest detection and identification, it is compared with the current mainstream two-stage and one-stage detection algorithms, respectively. Specifically, the second stage includes Faster R-CNN [16], FPN [33], Dynamic R-CNN [34], and Spare R-CNN [17]. These algorithms first scan potential objects on the feature map through a sliding window, then classify them, and return to the corresponding frame coordinates to detect the objects. The first stage includes RefineDet [35], YOLOv3 [36], SSD300 [32], PAA [37], TOOD [15], and YOLOX [14]. These methods directly regress the detected target category and location.  Table 1 shows the comparison results. The second-stage methods Faster R-CNN [16], FPN [33], Dynamic R-CNN [34], and Spare R-CNN [17] are superior to the first-stage detection methods RefineDet [35], YOLOv3 [36], and SSD300 [32]. The detection accuracy of YOLOX [14] is second only to the improved method in this paper. The improved method in this paper has higher detection accuracy than YOLOX, especially on small-scale targets.

### 4.5. Ablation Experiment

According to the ablation results in Table 2, an evaluation of each augmentation component on the IP102 dataset is shown. The baseline is YOLOX. RE means random erasing data enhancement, which can improve the robustness against image noise, e.g., partial occlusions and imperfect detections. The IN notes the improved neck. The improved YOLOX has achieved better results. It is proved that the algorithm proposed in this paper takes shallow information into account and further introduces dark2 to extract more robust fine-grained features, which is more conducive to the detection of small targets (AP_small_ increases 1.6%). A cross-scale fusion method is added, and the adaptive weight SUM is added to each fusion. As a result, the ablation experiments illustrate the evaluation of each augmentation component in our method.

### 4.6. Result Visualization

Figure 11 shows some results of this experiment, which intuitively reflects the effectiveness of the algorithm proposed in this paper. As can be seen from the figure, the target accounts for a large or small area of the picture, and all of them can correctly detect and identify the opposite category.

## 5. Conclusions

In this paper, the current pest identification methods are limited by the small dataset, which easily leads to the knowledge limitation and overfitting of model learning, the extracted features are too simple and not robust enough, and the generalization ability in actual scenes is insufficient. Taking YOLOX [14] as the framework, on this basis, the task of forest pest detection was improved. Firstly, aiming at the problem that there were few image data of real deep forest pests in the wild, we used Mosaic, Mixup, and random erasure to preprocess the data to prevent overfitting. Secondly, in order to extract fine-grained features [38], shallow information was introduced into the existing network architecture, and a two-way cross-scale feature fusion mechanism was adopted. The ablation experiment proved the rationality of each strategy of the improved method in this paper. The best performance on public datasets proved the effectiveness of this method. In the future, we will focus on the tiny model and transplant it to the handheld terminal.

## Figures and Tables

**Figure 1:** The framework of the algorithm in this paper.

**Figure 2:** Mosaic and mixup data enhancement visualization.

**Figure 3:** Network diagram of darknet-53.

**Figure 4:** Schematic diagram of focus.

**Figure 5:** Schematic diagram of Focus.

**Figure 6:** Schematic diagram of SPP structure.

**Figure 7:** Schematic diagram of the cross-scale fusion mode.

**Figure 8:** Model structure diagram of the head part.

**Figure 9:** Schematic diagram of the decoupled head.

**Figure 10:** Samples of partial categories of the dataset.

**Figure 11:** Sample detection results on the IP102 dataset.

**Algorithm 1:** Fusion.

**Table 1:** Average precision performance of state-of-the-art object detection methods under different IoU thresholds on IP102.

	AP_50_90_	AP_50_	AP_75_	AP_small_	AP_medium_	AP_large_
FPN	28.10	54.93	23.30	—	—	—
SSD300	21.49	47.21	16.57	—	—	—
RefineDet	22.84	49.01	16.82	—	—	—
YOLOv3	25.67	50.64	21.79	—	—	—
Faster R-CNN	28.4	48.0	30.2	17.8	29.0	29.4
PAA	25.2	42.7	26.1	18.6	27.1	26.1
Dynamic R-CNN	29.4	50.7	30.3	14.6	25.9	30.4
TOOD	26.5	43.9	28.7	19.0	28.3	27.4
Spare R-CNN	21.1	33.2	23.8	10.2	24.3	22.0
YOLOX	31.1	52.1	32.3	23.2	32.4	32.0
Improved YOLOX	32.4	53.6	33.4	24.8	33.5	32.9

**Table 2:** Evaluation of each augmentation component on IP102 datasets.

	AP_50_90_	AP_50_	AP_75_	AP_small_	AP_medium_	AP_large_
Baseline	31.1	52.1	32.3	23.2	32.4	32.0
Baseline + RE	31.8	52.9	32.7	23.4	32.9	32.1
Baseline + RE + IN (ours)	32.4	53.6	33.4	24.8	33.5	32.9

## Data Availability

The IP102 dataset used to support the findings of this study has been deposited in the PRCV2019 repository (DOI: 10.1109/CVPR.2019.00899).
